# Lightweight high-precision SAR ship detection method based on YOLOv7-LDS

**DOI:** 10.1371/journal.pone.0296992

**Published:** 2024-02-13

**Authors:** Shiliang Zhu, Min Miao

**Affiliations:** 1 School of Communication, Beijing Information Science and Technology University, Beijing, China; 2 Key Laboratory of the Ministry of Education for Optoelectronic Measurement Technology and Instrument, Beijing, China; Sichuan University, CHINA

## Abstract

The current challenges in Synthetic Aperture Radar (SAR) ship detection tasks revolve around handling significant variations in target sizes and managing high computational expenses, which hinder practical deployment on satellite or mobile airborne platforms. In response to these challenges, this research presents YOLOv7-LDS, a lightweight yet highly accurate SAR ship detection model built upon the YOLOv7 framework. In the core of YOLOv7-LDS’s architecture, we introduce a streamlined feature extraction network that strikes a delicate balance between detection precision and computational efficiency. This network is founded on Shufflenetv2 and incorporates Squeeze-and-Excitation (SE) attention mechanisms as its key elements. Additionally, in the Neck section, we introduce the Weighted Efficient Aggregation Network (DCW-ELAN), a fundamental feature extraction module that leverages Coordinate Attention (CA) and Depthwise Convolution (DWConv). This module efficiently aggregates features while preserving the ability to identify small-scale variations, ensuring top-quality feature extraction. Furthermore, we introduce a lightweight Spatial Pyramid Dilated Convolution Cross-Stage Partial Channel (LSPHDCCSPC) module. LSPHDCCSPC is a condensed version of the Spatial Pyramid Pooling Cross-Stage Partial Channel (SPPCSPC) module, incorporating Dilated Convolution (DConv) as a central component for extracting multi-scale information. The experimental results show that YOLOv7-LDS achieves a remarkable Mean Average Precision (mAP) of 99.1% and 95.8% on the SAR Ship Detection Dataset (SSDD) and the NWPU VHR-10 dataset with a parameter count (Params) of 3.4 million, a Giga Floating Point Operations Per Second (GFLOPs) of 6.1 and an Inference Time (IT) of 4.8 milliseconds. YOLOv7-LDS effectively strikes a fine balance between computational cost and detection performance, surpassing many of the current state-of-the-art object detection models. As a result, it offers a more resilient solution for maritime ship monitoring.

## 1. Introduction

The ocean economy is one of the key pillars supporting the development of human civilization in the new century [1]. However, maritime operations entail significant risks. Timely satellite-based observation to locate distressed ships for rescue or the utilization of mobile airborne equipment for surveying pirate ships are crucial tasks to ensure the safety of personnel. Therefore, researching efficient automated methods for detecting ships at sea holds significant practical engineering significance.

Synthetic Aperture Radar (SAR) imaging overcomes the drawbacks of optical imaging, which is susceptible to strong light and fog interference, allowing for uninterrupted observations around the clock. With the continuous advancement of SAR technology, it has greatly increased the success rate of maritime ship detection and rescue operations. However, SAR images captured by satellites or mobile airborne devices often contain background noise and interference from sea clutter. Additionally, the variability in shooting height and ship category leads to significant differences in ship pixel sizes within the images, presenting certain challenges in ship recognition and detection.

Traditional machine learning detection methods typically involve feature extraction using methods such as gradient direction histograms [2] and scale invariant feature transforms [3]. These extracted features are then input into classifiers like Support Vector Machine (SVM) [4] and iterators [5] for target detection and classification. The Constant False Alarm Rate (CFAR) algorithm [6] is the most widely used traditional detection method in SAR ship detection. However, CFAR requires setting thresholds based on the contrast between the target and background, which is subject to human expertise and specific scenarios. Traditional algorithms that rely on manual parameter adjustments struggle to adapt to the complex and dynamic scenes and significant variations in targets encountered in SAR ship image detection.

The rise of deep learning has propelled revolutionary advancements in the field of SAR ship detection. Compared to traditional target detection algorithms that rely on prior information, deep learning typically offers higher detection accuracy and robustness. Currently, SAR ship detection models based on deep learning can be broadly categorized into two types: two-stage detection and one-stage detection. Two-stage detection models divide the detection task into two stages: candidate region proposal and target regression. These models first generate candidate regions and then perform classification and localization within these regions. While these models often achieve high detection accuracy, as seen in classical algorithms like Regions Convolutional Neural Network (R-CNN) [7], Faster R-CNN [8], and Mask R-CNN [9], they tend to have a higher computational cost and slower detection speeds. One-stage algorithms, on the other hand, are end-to-end detection methods that directly produce output from input. Despite having relatively lower detection accuracy, they offer faster detection speeds. Examples of one-stage algorithms include the Single-Shot Multibox Detector (SSD) series [10] and the You Only Look Once (YOLO) series [11–17]. The YOLO series is currently the most popular one-stage object detection algorithm. In recent years, many researchers have proposed improvements based on the YOLO series to better suit the characteristics of SAR ship images, achieving outstanding detection accuracy and efficiency.

Li et al. [18] replaced the standard Convolution (Conv) in the YOLOv5 C3 module with deformable convolution, enhancing the model’s ability to extract global information by adjusting the sampling positions of pixels within the receptive field to adapt to changes in target scale. However, the use of deformable convolutions introduces a significant amount of additional computational complexity and parameter count. Ren et al. [19] employed MobileNetV3 [20], which incorporates Channel and Position Enhancement Attention (CPEA), as the backbone for YOLOv5l.This redesign aimed to reduce the model’s computational complexity and parameter count while improving the accuracy of target position information. Additionally, they incorporated Squeeze-and-Excitation (SE) attention mechanism [21] and added shallow pathways with more texture information in the multi-scale fusion nodes to enhance the model’s ability to extract features across various scales. Wang et al. [22] designed multi-scale convolution residual modules with rich hierarchical receptive fields and data augmentation blocks based on the transformer [23]. These modules were applied to the backbone network of YOLOX to enhance the model’s capability to capture global features and contextual information. Yu et al. [24] based on YOLOv5 introduced an improved Bidirectional Feature Pyramid Network (BIFPN) [25] to address the challenge of varying scales in SAR ship detection. They also added a Coordinate Attention (CA) [26] to the down-sampling modules of the backbone network to capture target position information. Su et al. [27] proposed a Spatial Information Integration Network (SII-Net) specifically designed for SAR ship detection. SII-Net integrates a Channel and Location Attention Mechanism (CLAM) and multiple pooling modules to obtain rich target position information. They also introduced interpolation pooling blocks to the backbone network’s output section to enhance the model’s sensitivity to small targets. Zhao et al. [28] introduced a preprocessing method tailored for SAR images to capture target edge information and reduce the impact of noise. This approach was applied to the input of YOLOv4-tiny to enhance the model’s sensitivity to small targets. Considering the background noise interference characteristic of SAR images, Zhang et al. [29] introduced a Frequency Attention Mechanism (FAM) in YOLOv5s to adaptively process frequency domain information and suppress sea clutter using captured frequency information.

While the aforementioned models have made significant strides in improving detection performance, they still come with a high computational cost. To strike a balance between model detection performance and lightweight design in SAR ship detection, ensuring excellent detection results on hardware-constrained mobile devices, this paper based on YOLOv7 propose a lightweight, high-precision SAR ship detection model (YOLOv7-LDS). The main contributions of YOLOv7-LDS are as follows:

1. Considering both detection accuracy and computational cost, we designed a light-weight network called SESNet, which serves as the backbone for YOLOv7-LDS. SESNet is a variant of ShuffleNetv2 that incorporates improvements such as SE attention mechanisms and Grouped Convolution (GConv). These introduced improvements effectively suppress background interference and overcome the limitations of complete channel isolation in Depthwise convolu-tions (DWConv).
2. In order to reduce computational costs and enhance sensitivity to target scale varia-tions, we made improvements to the Efficient Layer Aggregation Network (ELAN) within the neck module. These enhancements include substituting some standard convolutions with DWConv, refining convolution paths to improve scale adaptability, introducing a weighted channel connection method to optimize feature map fusion, and incorporating CA to precisely extract target position information. This culminated in the development of a weighted efficient aggregation network known as DCW-ELAN, based on CA and DWConv. Additionally, we replaced the SiLU activation function with Mish activation function [30] in the neck module and streamlined the Mixed Convolution Pooling down-sample module (MP) to enhance model efficiency.
3. To enhance the adaptability of the model to multi-scale variations in targets and further reduce computational costs, this paper introduces the Lightweight Spatial Pyramid Dilated Convolution Cross Stage Partial Channel module (LSPHDCCSPC). LSPHDCCSPC is a compressed version of the Spatial Pyramid Pooling Cross Stage Partial Channel (SPPCSPC) module, where Dilated Convolution (DConv) is introduced as the core component for extracting multi-scale information.

## 2 Overall architectures of the baseline and improved models

### 2.1 YOLOv7

YOLOv7 stands out as the most stable and impressive performer within the YOLO series. It excels in both speed and accuracy when compared to the currently popular YOLOv5, while surpassing YOLOv8 in terms of stability. The fundamental architecture of YOLOv7, as illustrated in Fig 1, primarily consists of four components: the input stage, the backbone, the neck, and the prediction head.

**Fig 1:** The overall architecture of YOLOv7.

YOLOv7 adopts the Mosaic data augmentation method introduced in YOLOv4 at the input stage. This involves randomly cropping and stitching four images to create a new composite image for training, enhancing dataset diversity and improving training efficiency. The backbone and neck primarily consist of CBS, ELAN, and MP. CBS is composed of cascaded Convolution layers, Batch Normalization layers (BN), and the SiLU activation function. ELAN comprises multiple cascaded CBS units, enhancing feature extraction by connecting the OFMs of each CBS. MP combines convolutional down-sampling and pooling down-sampling in parallel. At the junction between the backbone network’s tail and the neck, there is an SPPCSPC module used for extracting and fusing multi-scale information, consisting of multiple maximum pooling modules and a series of CBS for feature concatenation. Compared to the backbone network, the Neck section utilizes the ELAN-C module, includes an additional up-sampling module, and leverages the FPN+PAN structure for merging shallow and deep-level features, thereby extracting rich information. Compared to previous YOLO versions, the prediction head employs RepConv to increase feature information without adding complexity to inference computations.

It can be observed that the YOLOv7 model is a type of object detection model capable of effectively extracting feature information. Its widespread use of the multi-scale receptive field fusion method enables a high level of integration between the local and global information of objects. However, YOLOv7’s high computational complexity, extensive parameter count, and the inference power consumption on hardware pose limitations for its deployment in resource-constrained edge devices, such as maritime mobile airborne equipment or satellites. To efficiently utilize YOLOv7 on-edge devices, this paper has introduced lightweight improvements tailored for SAR image detection, resulting in the development of YOLOv7-LDS.

### 2.2 YOLOv7-LDS

The overall architecture of the YOLOv7-LDS object detection model is depicted in Fig 2. YOLOv7-LDS continues to employ the Mosaic data augmentation algorithm from YOLOv7 to enrich the dataset. The backbone network has been replaced with SESNet to significantly reduce the model’s computational complexity and parameter count. The basic component CBS in the neck has been substituted with CBM, which consists of Convolution, Batch Normalization (BN), and Mish activation functions cascaded together. A custom lightweight feature extraction module, DCW-LEAN, designed specifically for SAR images, has replaced the original ELAN-C module. The MP has been replaced with CBM(*K* = 3, *S* = 2), where K represents the convolution kernel size, and S denotes the stride. LSPHDCCSPC, which is lighter and excels in multi-scale feature extraction, has taken the place of SPPCSPC. The heavy RepConv blocks in the prediction head have been replaced with regular Conv(*K* = 3, *S* = 1).

The images to be examined contain ships of various scales, entering YOLOv7-LDS from the top of the backbone. Through convolution and down-sampling operations of multiple SESBlocks, feature maps {F1, F2, F3} are generated at large, medium, and small scales. These feature maps exhibit a gradual increase in semantic information and a corresponding decrease in detail information. F3, containing the highest semantic information, undergoes further processing through the LSPHDCCSPC module to extract features at more hierarchical scales, resulting in the formation of feature map F4. In the neck, {F1, F2, F4} undergo processing through the DCW-ELAN and CBM modules to extract more semantic information. Additionally, a fusion of detail and semantic information is achieved by concatenating with feature maps at different scales. The processed feature maps {F1’, F2’, F4’} generated by the neck are subsequently fed into small, medium, and large target detection heads, respectively. This allows for the capture of ships of different resolutions and sizes. Specifically, each detection head derives multiple anchor boxes of different sizes, generating candidate boxes on the image. This adaptive approach enables the model to accommodate ships with diverse aspect ratios. Finally, the Complete Intersection over Union (CIOU) and Non-Maximum Suppression (NMS) algorithms are applied to eliminate redundant candidate boxes, resulting in the most representative and final predicted boxes.

**Fig 2:** The overall architecture of YOLOv7-LDS.

## 3 Improved methodology

### 3.1 Shufflenetv2 and SESNet

Model lightweighting helps enhance its adaptability to various hardware platforms, while also reducing energy consumption and hardware resource requirements during runtime. Shufflenetv2 is a lightweight CNN model originally designed for image classification tasks. Due to its remarkably low parameter count and computational load, it is frequently employed as the backbone network in improved lightweight models for object detection [31, 32].

Fig 3illustrate the two primary building blocks of Shufflenetv2, namely, Shufflenetv2 Block1 and Shufflenetv2 Block2. Shufflenetv2 Block1 consists of two branches, where the left branch serves as a shortcut bypass, and the right branch represents the primary feature extraction path. The Input Feature Map (IFM) is initially split into two intermediate feature maps along the channels. One of these enters the right branch and undergoes feature extraction through Conv(*K* = 1, *S* = 1), DWConv(*K* = 3, *S* = 1), and Conv(*K* = 1, *S* = 1) modules. The other intermediate feature map directly enters the left branch and is concatenated with the output from the right branch. Subsequently, the concatenated feature map undergoes channel shuffling to shuffle the channel sequence, thereby preventing the repetition of feature extraction from the right branch by the next consecutive Shufflenetv2 Block1. Shufflenetv2 Block2 also comprises two branches, with the right branch structure closely resembling that of Shufflenetv2 Block1 but using DWConv(*K* = 3, *S* = 2). The left branch consists of DWConv(*K* = 3, *S* = 2) and Conv(*K* = 1, *S* = 1). While the IFM of Shufflenetv2 Block2 doesn’t need to be split, the intermediate feature maps from both the left and right branches require channel concatenation and shuffling to form the final output.

**Fig 3:** The fundamental building blocks of Shufflenetv2. (a) Shufflenetv2 Block1 (b) Shufflenetv2 Block2.

Compared to Conv, DWConv used in the ShufflenetV2 Block can significantly reduce computational complexity and the number of parameters. Fig 4(A) illustrates the working principle of Conv, where the weight filter dimensions are (*OC* = 4, *IC* = 4, *K* = 3, *K* = 3), the IFM dimensions are (*IC* = 4, *H* = h, *W* = w), and the OFM dimensions are (*OC*, *H*, *W*). Conv extracts information across the entire 3D space, encompassing inter-channel relationships and the feature map plane. The total computational load of Conv can be calculated by substituting the actual data from Fig 4(A) into the following formula:

OC×IC×K×K×H×W (1)

The total computation in Fig 4(A) amounts to 224×h×w. It’s worth noting that the computational complexity of the convolution layer is primarily focused on multiplication operations, and this formula only represents the number of multiplication operations. Fig 4(B) illustrates the operation of DWConv, where the dimensions of the weight filter are (*OC* = 1, *IC* = 4, *K* = 3, *K* = 3), while the dimensions of the input and OFMs are consistent with those inside Conv. DWConv extracts information only from the feature map plane, so the total computation in Fig 4(B) can be calculated using the following formula:

IC×K×K×H×W (2)

The total computation in Fig 4(B) amounts to 48×h×w. Compared to Conv, DWConv requires only 1/*OC* of the computation and parameter count. Despite its significantly reduced computational complexity and parameter count, DWConv does not extract inter-channel interactional information.

**Fig 4:** Working principles of different types of convolutions. (a) Conv (b)DWConv (c)GConv.

In this paper, to strike a balance between computational cost and detection accuracy, we propose the SES block based on the ShufflenetV2 block. Fig 5(A) and 5(B) illustrate two variations of the SES block: SES Block1 and SES Block2. The SES block replaces the DWConv in the ShufflenetV2 block with the more balanced group convolution (GConv) and adds an SE attention module after GConv to further enhance information exchange among feature channels and suppress background noise in SAR images. The operation of GConv is depicted in Fig 4(C), where the dimensions of the weight filters are (*OC* = 2, *IC* = 4, *K* = 3, *K* = 3), the IFM dimensions are (*IC* = 4, *H* = h, *W* = w), the OFM dimensions are (*OC*, *H*, *W*), and the grouping factor is *G* = 2. By employing the grouping factor, the output channels OC of the original Conv are reduced by half, and the weight filters and IFM channels *IC* are evenly divided into two groups. GConv independently calculates within each group, enabling it to extract information from the complete feature plane as well as partial interactions among channels. The total computational load can be calculated using the following formula:

$$G\times \frac{OC}{G}\times \frac{IC}{G}\times K\times K\times H\times W$$ (3)

**Fig 5:** The fundamental building blocks of SESNet. (a) SESNet Block1 (b) SESNet Block2.

The total computation in Fig 4(C) amounts to 48×h×w. Furthermore, as the value of *G* increases, the overall computation decreases, but the inter-channel information exchange diminishes, and vice versa. In equivalent configurations, the computation ratio between GConv and DWConv is *OC*/*G*:1. In this paper, different values of G are set based on the channel sizes in various layers of the SES Blocks, with larger channels corresponding to larger *G* values. The specific configurations can be found in Table 1.

**Table 1:** The configuration details for Shufflenetv2 and SESNet.

Shufflenetv2	Output channels	*G*	Repeat	SESNet	Output channels	*G*	Repeat
Input	3	-	-	Input	3	-	-
CBRM	24	-	-	CBRM	32	-	-
Block2	48	48	1	Block2	64	8	1
Block1	48	48	3	Block1	64	8	3
Block2	96	96	1	Block2	128	16	1
Block1	96	96	7	Block1	128	16	7
Block2	192	192	1	Block2	256	32	1
Block1	192	192	3	Block1	256	32	3

The structure of the SE Attention module, used to enhance inter-channel information exchange, is depicted in Fig 6 and consists of two stages: squeeze and excitation. In the squeeze stage, the IFM *X* undergoes global average pooling to obtain a feature vector *C1*, representing the channel dimension, with dimensions of c×1×1. In the excitation stage, this vector goes through a series of operations including fully connected layers (FC), ReLU, another FC layer and H_Sigmoid, facilitating inter-channel information exchange. This process yields a weighted factor vector *C2*. Finally, *C2* is multiplied channel-wise with *X* to generate an OFM *Y* that emphasizes target features, enhancing the interaction among channel information.

**Fig 6:** The structural design of the SE attention module.

Table 1 provides a detailed breakdown of the configuration information for SESNet, serving as the backbone network for YOLOv7-LDS, as well as the configuration information for the baseline model, Shufflenetv2. SESNet is comprised of SES blocks and CBRM modules. The CBRM modules consist of Conv(*S* = 3, *K* = 2), BN, ReLU and Max-Pooling. These modules serve as a preprocessing step on the original input images to reduce the complexity of subsequent computations. Additionally, the number of channels in each level of SESNet slightly differs from Shufflenetv2 to align channels between the shallow- level information in the backbone network and the deep-level information in the neck network. This alignment enhances the proportion of fine-grained details required for small target detection. It’s worth noting that R represents the number of times a particular module or component is repeated within the corresponding model.

### 3.2 Lightweight enhancements of the neck and DCW-ELAN module

To further reduce the overall computational cost and enhance object detection capabilities, this paper has undertaken lightweight enhancements to the ELAN-C module within the Neck section. These enhancements include the introduction of DWConv, the incorporation of a CA module, and the implementation of a weighted feature fusion mechanism. Consequently, this results in the creation of the DCW-ELAN module, which possesses adaptive multi-scale feature extraction capabilities and the ability to capture rich positional information. Additionally, this paper has opted to discard the structurally complex MP in favor of directly utilizing CBM(*K* = 3, *S* = 2) as the down-sampling module.

Fig 7 depict the structures of ELAN-C and DCW-ELAN, respectively. In comparison to ELAN-C, the feature extraction portion of DCW-ELAN comprises only 4 modules: 2 CBM(*K* = 1, *S* = 1) and 2 DBM(*K* = 3, *S* = 1). This not only preserves more detailed information but also reduces the computational complexity and parameter count of the model. The CBM consists of cascaded the Conv, BN, and Mish activation function, while the DBM is composed of DWConv, BN, and Mish activation function. The Mish activation function has a lower bound but no upper bound. When its input approaches extremes, the gradient tends to be close to 1. This effectively mitigates the slow convergence issue caused by zero gradients during network training. Furthermore, it exhibits better noise suppression characteristics compared to SiLU. Its mathematical expression is as follows:

$$Mish=x\times tanh(ln(1+e^{x}))$$ (4)

**Fig 7:** The core feature extraction modules of the Neck network. (a) Structure of ELAN-C (b) Structure of DCW-ELAN.

Traditional feature fusion methods often involve a simple concatenation of feature maps from different scales. However, it’s essential to recognize that feature maps from different scales may contribute differently to subsequent information extraction and could even lead to information interference. Therefore, in the feature fusion component of DCW-ELAN, a normalized feature-weighted fusion approach is employed. This method assigns varying weights to feature maps from different scales before fusing them, mitigating the aforementioned issues. The formula for weighted fusion is expressed as follows:

$$W_{i}=\frac{I_{i}}{\sum_{i=1}^{4}I_{i}+e}$$ (5)

$$Y=Concat(W_{1}\times X_{1}+W_{2}\times X_{2}+W_{3}\times X_{3}+W_{4}\times X_{4})$$ (6)

In this formula, (*X1*, *X2*, *X3*, *X4*) represent four sets of IFMs at different scales in DCW-ELAN, while *Y* is the output of the WConcat component. *W*_*i*_ represents the weights corresponding to each set of input features, and the corresponding *I*_*i*_ is a set of trainable parameters with an initial value of 1. The e represents the initial learning rate, which is set to 0.0001 to prevent numerical instability during computations. Following the fusion stage, the CA attention mechanism module at the end of DCW-ELAN has the ability to suppress interference from sea clutter in complex environments where SAR ships are located, capture positional information between targets, and enhance the model’s ability to detect targets of various scales.

Fig 8 illustrates the structure of the CA module. Firstly, for the IFM *X* with dimensions (*C*, *H*, *W*), global average pooling is applied along the horizontal and vertical directions, compressing it into two vectors with dimensions (*C*, *H*, 1) for the vertical direction denoted as *x*1, and (*C*, 1, *W*) for the horizontal direction denoted as *x*2. Next, *x*1 and *x*2 are concatenated sequentially and then processed through Concatenation, CBS(*S* = 1, *K* = 1), and Split operations to obtain enhanced directional vectors, *x*1’ and *x*2’. Subsequently, *x*1’ and *x*2’ each go through Conv(*K* = 1, *S* = 1) and the sigmoid activation function, resulting in perception feature map vectors *x*1’’ and *x*2’’ representing horizontal and vertical distance information, respectively. Finally, the IFM *X* is multiplied sequentially with *x*1’’ and *x*2’’ to obtain the ultimate OFM *Y* containing spatial positional information.

**Fig 8:** The structural design of the CA module.

### 3.3 LSPDCCSPC

The original SPPCSPC structure in YOLOv7 is complex and redundant, requiring multiple cascading CBS and parallel large receptive field maximum pooling operations to extract multi-scale feature information. This complexity imposes a high computational cost on the model. To reduce the computational cost, eliminate the information redundancy caused by multiple cascading CBS, and achieve a more coherent extraction of multi-scale feature information, we purpose the LSPDCCSPC module. Fig 9 illustrate the architectures of SPPCSPC and LSPDCCSPC. The LSPDCCSPC module removes redundant convolution components from the original SPPCSPC module and replaces the parallel large receptive field maximum pooling with cascading mixed DConv.

**Fig 9:** The Multi-scale feature capture module structure. (a) SPPCSPC (b) LSPDCCSPC.

While dilated convolutions may introduce some additional computational complexity and parameters, maximum pooling compresses all values within each receptive field window into a single maximum value, leading to information loss, particularly when using larger receptive fields. DConv is helpful in preserving more of the original feature information and extracting inter-channel interactions. However, simply replacing consistent receptive field dilated convolutions in a parallel Max-Pooling structure may result in sparse sampling points, as shown in Fig 10(A). Therefore, we drew inspiration from the pooling structure of SPPF and adopted a cascading approach that combines dilated convolutions with different dilation rates to fill in the sampling gaps created by the parallel structure, as illustrated in Fig 10(B). This approach helps maintain sampling density and enhances the efficiency of information capture.

**Fig 10:** Illustration of the receptive field for a cascade of three K = 3 dilated convolution modules. (a) When all dilated convolution modules have an expansion factor of 2 (b) When the expansion factors of the dilated convolution modules incrementally increase, with values of 1, 2, and 3, respectively.

In the LSPDCCSPC module, the IFM *X* initially passes through the SPPCSPC module and then branches into two parallel paths, each going through a CBM(*S* = 1, *K* = 1) to form *X*1 and *X*2, respectively. To reduce subsequent computational complexity and the number of parameters, the channel dimensions of *X*1 and *X*2 are compressed to half of the original IFM *X*. Next, *X*1 enters the cascading mixed dilated convolution module for the extraction of multi-scale feature information. These multi-scale feature maps, along with *X*2 after concatenation, are fused through CBS(*S* = 1, *K* = 1) to form *X*3. Finally, *X* and *X*3 are concatenated and subsequently fused through CBS(*S* = 1, *K* = 1) to generate the final OFM *Y*. While the LSPDCCSPC module incorporates DConv, which may increase the computational load and the number of parameters, other components and the channel dimensions are relatively reduced. Consequently, the LSPDCCSPC module remains more lightweight than SPPCSPC while offering enhanced feature extraction capabilities.

## 4 Experiment

### 4.1 Experimental environment

All experiments in this paper were conducted in an environment consisting of Ubuntu 20.04, PyTorch 2.0.0, CUDA 11.8, Python 3.8, an NVIDIA RTX 4090 GPU with 24GB VRAM, and a 12 vCPU Intel(R) Xeon(R) Platinum 8352V CPU @ 2.10GHz.

### 4.2 Dataset and experimental setup

To validate the effectiveness of YOLOv7-LDS, we utilized the publicly available SAR Ship Detection Dataset (SSDD) [33]. This dataset comprises SAR images captured by the RadarSat-2, Terra, and SAR-XSentinel-1 satellites, encompassing coastal and nearshore backgrounds. It contains a total of 1160 images and 2456 object ships with varying scales. The visual representation in Fig 11(A) and 11(B) illustrates the statistical information of the ship dataset. It is evident that the SSDD covers a wide range of target scales, with a particular focus on the challenging category of small targets that are typically harder to detect. Additionally, this study introduces the NWPU VHR-10 optical remote sensing object detection dataset, publicly released by Northwestern Polytechnical University [34–36], to further validate the universality and robustness of YOLOv7-LDS. The dataset comprises 650 positive sample images, 150 negative sample images, 3775 object instances, and spans across 10. categories: airplane, ship, storage tank, baseball diamond, tennis court, basketball court, ground track field, harbor, bridge, and vehicle. Notably, 52 images within the dataset contain instances of the ship category along with other categories. Statistical information for the NWPU VHR-10 dataset is presented in Figs 11(C)–12(D). It is evident that the NWPU VHR-10 dataset covers a wide range of target scales, although a considerable proportion of targets are of smaller sizes.

**Fig 11:** Visualization of SSDD and NWPU VHR-10 object statistics, which darker colors indicate a higher number of target instances. (a) Schematic representation of the distribution of target instance center points of SSDD (b) Schematic representation of the distribution of target instance sizes of SSDD (c) Schematic representation of the distribution of target instance center points of NWPU VHR-10 (d) Schematic representation of the distribution of target instance sizes of NWPU VHR-10.

**Fig 12:** Introducing an attention mechanism for visualizing heatmap results of the model’s detection outcomes. (a) Ground truth bounding box label map for the targets (b) Without the introduction of an attention mechanism (c) Incorporating the SE attention mechanism (d) Incorporating the CA mechanism (e) Simultaneously introducing both SE and CA attention mechanisms. Reprinted from [33] under the Apache license and CC BY 4.0, with permission from Tianwen Zhang, original copyright 2021.

In this study, we randomly divided the SSDD into training and testing sets in an 8:2 ratio. We employed the Stochastic Gradient Descent (SGD) optimizer to update model parameters, with an initial learning rate of 0.01. The learning rate was adjusted using the cosine annealing algorithm until the end of training. Our choice of loss function was CIOU, and we applied NMS as the standard. Input image resolutions were standardized to 640×640, with a batch size of 32 and training conducted over 400 epochs. We also utilized caching to expedite training speed. During the image preprocessing phase, we applied Mosaic for data augmentation.

For the SSDD and NWPU VHR-10 datasets, the model parameters are updated using the Stochastic Gradient Descent (SGD) optimizer and the Adaptive Moment Estimation (Adam) optimizer, respectively. The initial learning rate is set to 0.01. The learning rate was adjusted using the cosine annealing algorithm until the end of training. Our choice of loss function was CIOU, and we applied NMS as the standard. The input image resolution is standardized to 640×640, and the batch size is set to 32. The training epochs for the SSDD and NWPU VHR-10 datasets are 400 and 1000, respectively. The ratio of the training set to the test set is 8:2.

### 4.3 Performance metrics

In this paper, a comprehensive set of evaluation metrics is utilized to assess the performance of the ship detection model. These metrics include Precision (P), Recall (R), mean Average Precision (mAP) at IOU = 0.5, Inference Time (IT), Parameters (Params), and Giga Floating Point Operations Per second (GFLOPs). Among these, IT, Params, and GFLOPs reflect the model’s lightweight characteristics, while P, R, and mAP reflect its detection capabilities. P, R, and mAP can be calculated using the following formulas:

$$P=\frac{TP}{TP+FP}$$ (7)

$$R=\frac{TP}{TP+FN}$$ (8)

$$mAP=\int_{0}^{1}P(R)dR$$ (9)

Here, TP represents the number of correctly detected ships, FP represents the number of misclassified ships, and FN represents the number of missed ships.

### 4.4 Ablation

In order to verify the effectiveness of each proposed improvement module, a series of ablation experiments are conducted in this paper for comparative analysis. The results are presented in Table 2. To ensure the accuracy and fairness of the experiments, we used the same hyperparameters and datasets during the training process.

**Table 2:** Ablation experiments on SSDD.

Experiment	Model	P%	R%	mAP%	Params(M)	GFLOPs	IT(ms)
A	YOLOv7	97.9	95.4	98.9	37.2	104.5	7.9
B	YOLOv7+SESNet	97.4	95.4	98.8	23.1	37.4	6.3
C	YOLOv7+CDELAN	97.1	97.1	98.7	23.6	77.5	6.7
D	YOLOv7+LSPDCCSPC	96.4	95.1	98.5	30.1	98.8	6.5
E	YOLOv7+SESNet+CDELAN	96.3	94.6	98.4	9.7	11.1	5.1
F	YOLOv7+SESNet+CDELAN+LSPDCCSC (**YOLOv7-LDS**)	97.7	96.6	99.1	3.4	6.1	4.8
G	YOLOv7+Shufflenetv2+CDELAN+ LSPDCCSPC	97.2	95.2	98.2	3.2	5.4	4.5

Experiment A presents the test results of YOLOv7 on SSDD, achieving P, R, and mAP of 97.9%, 95.4%, and 98.9%, respectively. However, YOLOv7 comes with a high computational cost, having a model Params(M) of 37.2, a GFLOPs of 104.5, and an IT of 7.9 ms.

Experiment B showcases the results of using SESNet as the backbone network for YOLOv7. The results demonstrate a successful reduction in computational cost while maintaining high detection performance. In this experiment, P, R, and mAP are similar to those in Experiment A, with Params(M) and GFLOPs reduced by 37.9% and 64.2%, respectively. Additionally, the IT is reduced by 1.6 ms.

Experiment C reveals the results of lightweight improvements made to the neck network of YOLOv7. In the neck network, ELAN is replaced by DCW-ELAN, CBS is substituted with CBM, and CBM (S = 3, K = 2) is used instead of MP. Compared to Experiment A, the mAP remains similar, P decreases by 0.8%, but R improves by 1.7%. Moreover, Params(M), GFLOPs, and IT are reduced by 36.6%, 25.8%, and 1.2 ms, respectively.

Experiment D presents the results of replacing the SPPCSPC modules in YOLOv7 with lightweight LSPDCCSPC modules. Compared to Experiment A, Params(M), GFLOPs, and IT are reduced by 19.0%, 5.4%, and 1.4 ms, respectively. However, P, R, and mAP decreased by 1.5%, 0.3%, and 0.4%, respectively. SPDCCSPC is not suitable for deep and complex models like YOLOv7 that heavily rely on Conv(K>3). This is because at the end of the backbone network, a significant amount of semantic information between channels has already been extracted, resulting in a reduction of detailed information. In this scenario, using max pooling, which does not extract channel information, would yield better detection results compared to using dilated convolutions.

Experiment E demonstrates simultaneous lightweight improvements to the backbone and neck networks of YOLOv7, combining the enhancements from Experiments B and C. In this experiment, Params(M) and GFLOPs are reduced to 9.7 and 11.1, respectively, compared to Experiment A. Additionally, IT is reduced by 2.8 ms. However, the dual lightweight approach leads to a decrease in detection performance, with P, R, and mAP dropping by 1.6%, 0.8%, and 0.5%, respectively.

Experiment F, built upon Experiment E, continues to enhance feature extraction capabilities by replacing the original SPPCSPC modules with LSPDCCSPC, resulting in the YOLOv7-LDS model. YOLOv7-LDS achieves P, R, and mAP values of 97.7%, 96.6%, and 99.1%, respectively, slightly outperforming YOLOv7 in overall detection capability. Furthermore, YOLOv7-LDS’s Params(M), GFLOPs, and IT are significantly lower, decreasing by 90.8%, 94.1%, and 3.1 ms, respectively, compared to YOLOv7. In comparison to Experiment D, this experiment yields better results due to the weaker channel feature extraction of SESNet and DCELAN, which LSPDCCSPC addresses by using dilated convolutions to compensate for pooling.

Experiment G assesses the performance of using the improved Shufflenetv2 as the backbone for YOLOv7-LDS and compares it to SESNet. The results show P, R, and mAP values of 97.2%, 95.2%, and 98.2%, respectively, with a slight decrease compared to Experiment F. Furthermore, there is little difference in computational cost and IT between the two.

### 4.5 Visualization of the impact of attention and detection results

To enhance the sensitivity of the model to the target objects, this paper embedded SE and CA mechanisms separately into the model’s backbone SESBlock and neck DCW-ELAN. Fig 12 presents the visual results of how SE and CA mechanisms influence the model’s attention. In the heatmaps, deeper shades of blue represent lower attention from the model to that specific target region, while deeper shades of red indicate higher attention. When attention mechanisms are not introduced, the model focuses on the target ships, but the red areas on the ships are not sufficiently deep, indicating relatively scattered attention. Additionally, the model shows interest in the coastline at the top right corner, resulting in red regions. With the introduction of the SE attention mechanism, the model shifts its focus away from the top right coastline, and the red regions on the ships become more concentrated. When the CA mechanism is introduced, the model again shifts its focus away from the top right coastline but renews its attention to the left coastline, resulting in deeper red regions on the ships. When both attention mechanisms are combined, the model generates eight major red temperature points, precisely aligning with each of the target ships. This outcome demonstrates that the combination of SE and CA mechanisms significantly enhances the model’s focus and detection performance on the targets.

To intuitively observe the detection performance of YOLOv7-LDS, Fig 13 illustrates the detection results of YOLOv7-LDS in five typical challenging scenarios from SSDD, along with corresponding ground truth horizontal bounding box annotations. The upper half displays the real box annotations, while the lower half shows YOLOv7-LDS’s detection results. In all these challenging scenarios, YOLOv7-LDS exhibits excellent detection performance, accurately annotating real ships with high confidence, demonstrating the robustness and effectiveness of YOLOv7-LDS.

**Fig 13:** LHSSNet’s ships detection results for five typical scenarios on SSDD dataset. (a) Scene with boats of varying sizes anchored along the shore (b) Scene where boats are surrounded by coastal structures (c) Detection scenario disrupted by small islands with textures similar to boats (d) More complex scene with coastal areas and islands as background interference, and smaller boats to be detected (e) Detecting scenarios of small ships with a significant amount of speckle noise, and where there is significant variability in the scale of the ships. Reprinted from [33] under the Apache license and CC BY 4.0, with permission from Tianwen Zhang, original copyright 2021.

Furthermore, Fig 14 showcases partial detection results of YOLOv7-LDS on the NWPU VHR-10 dataset along with corresponding ground truth horizontal bounding box annotations. The upper section displays annotations of actual bounding boxes, while the lower section presents the detection results of YOLOv7-LDS. The four scenarios depicted include: the first scenario with ships and other small targets, the second scenario illustrating variations in target scales, the third scenario featuring densely arranged aircraft for detection, and the fourth scenario highlighting the challenges of detecting small-sized target vehicles amid a background with numerous distracting objects. YOLOv7-LDS consistently demonstrates accurate target detection across these diverse scenarios.

**Fig 14:** LHSSNet’s remote sensing multi-category detection results on NWPU VHR-10 dataset. Reprinted from [34] under the CC BY license, with permission from Peicheng Zhou, original copyright 2023.

### 4.6 Comparisons with the state-of-the-art

This paper compared YOLOv7-LDS with eight different state-of-the-art lightweight object detection models, including Faster R-CNN, LPEDet [37], Cascade R-CNN [38], CRAS-YOLO [39], YOLOv4-tiny, YOLOv5s, YOLOv7-tiny, and LMSD-YOLO [40]. Table 3 presents the mAP, Params(M), GFLOPs, and IT of these models. It can be observed that YOLOv7-LDS achieves a mAP only 0.4% higher than CRAS-YOLO, but its Params(M), GFLOPs, and IT are approximately 33.0%, 30.9%, and 60.8% lower than YOLOv7-LDS, respectively. Additionally, although YOLOv7-LDS’s inference speed is slightly inferior to YOLO-tiny, its mAP is 1% higher, and Params(M) and GFLOPs are approximately 57% and 46.9% of YOLO-tiny, respectively. In comparison to other models, YOLOv7-LDS outperforms them in various performance metrics. In summary, YOLOv7-LDS strikes a good balance between accuracy and computational cost, making it suitable for resource-constrained maritime SAR ship detection systems.

**Table 3:** The detection results of YOLOv7-LDS and other state-of-the-art detectors on SSDD.

Model	mAP%	Params(M)	GFLOPs	IT(ms)
YOLOv7-LDS	99.1	3.4	6.1	4.8
YOLOv7-tiny	98.1	6.0	13.0	4.6
YOLOv5s	97.9	7.2	15.8	5.1
Yolov4-tiny	97.3	5.9	16.1	3.8
LMSDYOLO [40]	98.0	3.5	6.6	14.6
LPEDet [37]	97.4	5.7	18.4	7.0
Faster R-CNN	96.4	41.1	91.4	45.4
Cascade R-CNN [38]	96.8	69.1	119.0	65.56
CRAS-YOLO [39]	98.7	10.3	19.7	7.9

In addition, to further demonstrate that YOLOv7-LDS is a competent object detection model, this study compares it with YOLOv4-tiny, YOLOv5s, YOLOv7-tiny, HFPNet [41], Ran et al. [42], and Shen et al. [43] models on the NWPU VHR-10 dataset. The comparative results on this dataset are summarized in Table 4. In terms of mAP, YOLOv7-LDS ranks second, only 0.7% lower than YOLOv7-tiny; in Params(M), YOLOv7-LDS performs optimally, with an 8.1% reduction compared to the model based on the YOLOv8n improvement by Shen et al. [43]; in terms of GFLOPs, YOLOv7-LDS is only 24.4% higher than the model with the lowest computational complexity, Ran et al. [42]; in terms of IT, YOLOv7-LDS remains slower than YOLOv7-tiny and YOLOv4-tiny.

**Table 4:** The detection results of YOLOv7-LDS and other state-of-the-art detectors on NWPU VHR-10 dataset.

Model	mAP%	Params(M)	GFLOPs	IT(ms)
YOLOv7-LDS	95.8	3.4	6.1	4.8
YOLOv7-tiny	96.5	6.0	13.0	4.6
YOLOv5s	95.3	7.2	15.8	5.1
YOLOv4-tiny	93.0	5.9	16.1	3.8
HFPNet [41]	95.3	15.2	24.3	20.0
Ran et al. [42]	94.4	5.1	4.9	-
Shen et al. [43]	91.2	3.7	10.2	18.4

### 4.7 Comparison of YOLOv7-LDS with classical traditional object detection algorithms

Some traditional feature extraction algorithms, such as Scale Invariant Feature Transform (SIFT) [44, 45] and Histogram of Oriented Gradients (HOG) [46], are effective in capturing features of ship targets. Therefore, we extract partial images from the original feature map and use SIFT/HOG for feature extraction on these images. The extracted features are then input into a combination algorithm of SVM and NMS to generate prediction boxes for ship detection.

As SSDD lacks negative samples, we use the original training set images of SSDD as positive samples and segment some backgrounds from the training set images as negative samples, maintaining a ratio of 1:1 between positive and negative samples. However, these two traditional methods heavily rely on manual settings of detection boxes and detection image sizes. In addition, the inference speed fluctuates significantly with changes in the size of the images to be detected. To accommodate traditional methods, we intentionally standardized the resolution of training and testing images to 160×160. The test results, as shown in Table 5, indicate a certain gap in detection capabilities between traditional methods and YOLOv7-LDS. Compared to YOLO-LDS, their differences in precision (P), recall (R), and balanced F1 Score are 17.2%/21.9%, 29.0%/19.1%, and 27.0%/18.7%, respectively. Moreover, they exhibit extremely slow inference speeds, with inference times using CPU being 5.33s/1.02s, while YOLOv7-LDS takes only 0.17s, resulting in a difference of 31.4x/6.0x. F1 is the harmonic mean of precision and recall, and its expression is as follows:

$$F1=2\times \frac{P\times R}{P+R}$$ (10)

Fig 15 presents visual results of the detection for these three methods. In scenarios with minimal background noise interference, all three methods can relatively accurately detect ships. However, there is a center region offset in SIFT detection. In scenarios with strong background speckle noise interference, SIFT and HOG methods exhibit both missed detections and false positives, indicating significant interference from speckle noise on traditional algorithms. Nevertheless, YOLOv7-LDS continues to effectively detect ships. Additionally, the prediction boxes generated by traditional algorithms have a larger range, while those generated by YOLOv7-LDS are more focused on the target.

**Fig 15:** Visual comparison results between YOLOv7-LDS and classical traditional object detection algorithms, where the images processed by traditional algorithms underwent Gaussian filtering preprocessing. (a) Actual object annotation results (b) SIFT detection results (c) HOG detection results (d) YOLOv7-LDS detection results. Reprinted from [33] under the Apache license and CC BY 4.0, with permission from Tianwen Zhang, original copyright 2021.

**Table 5:** The detection results of YOLOv7-LDS and traditional algorithms.

Model	P%	R%	F1	IT(s)
SIFT+SVM+NMS	73.8	49.2	59.1	5.33
HOG+SVM+NMS	78.5	59.1	67.4	1.02
YOLOv7-LDS	95.7	78.2	86.1	0.17

## 5 Conclusion

A lightweight and easily deployable high-precision ship detection model is crucial for maritime operations. It can play a vital role in tasks such as identifying distressed vessels, preventing pirate ships, or tracking suspicious vessels during long-term operations at sea using high-altitude drones or mobile satellite equipment. Especially in the case of high-altitude, long-duration drone operations, managing energy consumption is a key challenge. Therefore, achieving high-precision ship detection with low-power hardware platforms is of utmost importance. Additionally, Synthetic Aperture Radar (SAR) technology allows for ship detection imaging in all weather conditions. In light of these considerations, this paper proposes a lightweight and high-precision SAR ship target detection model named YOLOv7-LDS. YOLOv7-LDS is a lightweight improvement upon the powerful YOLOv7 model.

The backbone network of YOLOv7-LDS is an enhanced version of Shufflenetv2, referred to as SESNet. SESNet incorporates SE and GConv enhancements to balance detection accuracy and computational cost. Experimental results show that when SESNet is used as the backbone network for YOLOv7-LDS, it improves mAP by 0.9% compared to using the original Shufflenetv2, with only a minor increase in model parameters, GFLOPs, and IT. YOLOv7-LDS’s Neck module introduces an DCW-ELAN that utilizes DWConv, CA, and a weighted feature fusion mechanism. This preserves more fine-grained details required for detecting small targets and adjusts the influence weights of different-scale features on target detection. It achieves this while reducing computational cost and maintaining efficient feature extraction. This paper performs lightweight and enhanced improvements on YOLOv7’s SPPCSPC to create LSPDCCSPC. LSPDCCSPC replaces the original parallel pooling module with a cascade of dilated convolution layers with increasing dilation rates. This reduces the redundancy in the channel concatenation structure of SPPCSPC.

On SSDD, extensive ablation experiments, heatmap visualization, detection visualization, and comparisons with other state-of-the-art models are conducted for YOLOv7-LDS. Results demonstrate that the proposed improvements significantly enhance the model’s overall detection capabilities while striking a good balance between computational cost and detection accuracy. Specifically, YOLOv7-LDS achieves a mAP of 99.1%, with 3.4M Params, 6.1 GFLOPs, and an IT of 4.8 ms. Heatmap visualization results indicate that the introduction of SE and CA modules allows the model to better focus on the location of the target to be detected. Detection visualization confirms that YOLOv7-LDS performs well in various challenging detection scenarios. When compared to several state-of-the-art models, YOLOv7-LDS consistently ranks at the forefront, further proving its effectiveness for maritime operations. We also validated the YOLOv7-LDS model on the NWPU VHR-10 dataset, achieving a mAP of 95.8%. Its overall performance surpasses most state-of-the-art models currently available. Furthermore, the favorable comparison results with classical traditional algorithms further underscore the superiority of YOLOv7-LDS. Furthermore, existing research has confirmed that the fusion of SAR, optical, and thermal images can enhance the feature representation capability of targets [47, 48]. We plan to make corresponding improvements to YOLOv7-LDS for multimodal detection in the future, combining different imaging features to enhance the model’s detection capabilities for targets in complex environments, not limited to ship detection alone.
